The article "Investigation on Immune-Related Protein (Heat Shock Proteins and Metallothionein) Gene Expression Changes and Liver Histopathology in Cadmium-Stressed Fish" was retracted in 2024. Reasons: signs of a paper mill; suspected computer-generated content; unreliable results or conclusions; concerns about the data.

# Investigation on Immune-Related Protein (Heat Shock Proteins and Metallothionein) Gene Expression Changes and Liver Histopathology in Cadmium-Stressed Fish

**DOI:** 10.1155/2022/2075791

**Published:** 2022-08-03

**Authors:** Ghazala Jabeen, Sarwat Ishaq, Mateen Arshad, Shafaq Fatima, Zakia Kanwal, Farah Ali

**Affiliations:** ^1^Department of Zoology, Lahore College for Women University, Lahore, Pakistan; ^2^Department of Theriogenology, Faculty of Veterinary and Animal Sciences, Islamia University Bahawalpur, Pakistan

## Abstract

Heat shock proteins (HSP) are highly conserved in their structure and released in case of stress. Increased metallothionein (MT) synthesis is associated with increased capacity for binding heavy metals. Healthy juveniles of grass carp were exposed to sublethal dose (1.495 mg L^−1^) of cadmium for 28 days. Simultaneously, a control group was also run to compare difference of total RNA expression levels in cadmium-treated and control groups. The cadmium levels in the tissues of treated fish recorded were 1.78 ± 0.10 mg L^−1^, 1.60 ± 0.04 mg L^−1^, and 2.00 ± 0.05 mg L^−1^, respectively. Several histological alterations including edema, hemorrhage, dilated sinusoids, hypertrophy, hyperplasia, congestion of central vein, and nuclear alterations were observed in cadmium-exposed fish. Stress gene (metallothionein and heat shock proteins) mRNA transcription levels were studied by mRNA extraction and cDNA preparation by using PCR. The expression level of heat shock protein gene was higher as compared to metallothionein and beta-2-microglobulin gene after cadmium exposure. This study reports various stress-related immune-responsive changes of immune proteins, heat shock proteins, metallothionein, and histopathological changes in fish due to cadmium toxicity that make the fish immunocompromised which may be considered as the biomarkers of cadmium toxicity in other experimental species.

## 1. Introduction

Heat shock proteins (HSP) are involved in signaling network to reprogram gene transcription, folding and unfolding of proteins, changes in mRNA translation, and degradation of misfolded proteins to ensure protein quality control [1]. Heat shock proteins act as the first line of protection for cells exposed to stressful conditions. They maintain the cell integrity and functionality of the cell signaling pathways critical for regular cell function and cell survival. Because these proteins are induced in the presence of stressors like hot and cold temperature shock, heavy metal toxicity, free radicals, oxidants, toxins, and viruses [2]. HSP70 is an inducible protein and considered major protein of HSP family. HSP performed housekeeping functions and are molecular chaperones in cell.

Metallothioneins are cytosolic protein that conserved in cysteinyl residues. These residues are arranged in two thiol-rich sites with basic amino acids (lysine and arginine) and help to attach, transport, and store heavy metals through thiolate bonding [3]. Expression changes of metallothioneins gene are used as biomarker in fish for detecting water pollution due to heavy metals [4]. Metallothioneins are low molecular weight proteins produced in the presence of divalent ions of cadmium and attach with it for lower the toxicity. But when cadmium is present in high concentration and overcome on detoxification system of metallothionein, then cadmium toxicity effect will be increased [5, 6].

Cadmium is a nonessential element for organisms and considered most toxic heavy metal. Big industries' wastewater has high concentration of cadmium that mixes with river water [7]. Structural and functional changes occur in fish organs due to cadmium accumulation. Cadmium higher concentration was recorded in fish liver and kidney [8]. Heavy metals cadmium, mercury, copper, and zinc induce metallothionein. These are small proteins containing ~7 kDa weight. Cadmium accumulates in liver tissues and causes structural and functional alteration in liver tissues like congestion, blood vessel damages, hepatocyte degeneration, pancreatic cell necrosis, and change in the fats of peripancreatic hepatocytes [9]. Biomarkers are used for indication of histopathological changes and water pollutants. Histological biomarkers are related with the stress biomarkers. Metabolic activation initiated in the presence of many pollutants that induce cellular changes. Several xenobiotics mechanism of action produced specific enzymes that induce metabolic changes, cellular intoxication, cellular death, and cellular necrosis [10]. HSP70 has been sequenced in tilapia [11], rainbow trout [12] and zebrafish [13]. The expression of HSP70 is increased in the presence of proteotoxic environmental stressors.

Cadmium is a hazardous, toxic, and inessential metal that poses a serious health risk for aquatic biota and humans. The potential causes of cadmium toxicity are agricultural and industrial sources leading to the contamination of food and water [14]. The environmental cadmium exposure may be a risk factor due to the toxic impact on the liver and kidneys. These organs are more vulnerable to cadmium's toxicity due to their synthesis ability to produce Cd-inducible proteins, metallothionein proteins that protect the cells [15]. Cadmium exposure causes disorders in metabolic functions, reproduction, growth, developmental anomalies, and immunity suppression due to the accumulation of cadmium in the vital body organs [16–18]. Aquatic ecosystem contamination has proved to be a great threat to natural communities and ecosystem. Cadmium exposure instigates the histopathological changes in vital tissues of animals due to bioaccumulation of metal in the cells [19]. The liver is considered as the dynamic multifunctional organ involved in the metabolism and detoxification of the toxic metals due to the presence of immune-related cells like lymphocytes, neutrophils, kupffer cells, and macrophages [17, 18, 20]. Therefore, the objectives of the current study were to investigate the impact of cadmium on fish health, changes in tissue structure and mRNA expression levels of the immune-related proteins like metallothionein (MT), heat shock proteins (HSP), and beta-2-microglobulin (B2M) genes in control and cadmium-treated liver tissues by using PCR.

## 2. Materials and Methods

### 2.1. Experimental Design

A total of 100 freshwater fish (*Ctenopharyngodon idella*) weighing about 6.20 ± 2.38 g and measuring 9.60 ± 1.84 cm in length were collected in plastic bags supplemented with appropriate oxygen from a public fish seed hatchery. After acclimatization, fish were divided into two groups, control group (normal tap water with continuous aeration) and treatment group subjected to sublethal concentration (1/10 LC_50_, 1.495 mg L^−1^) of cadmium based on predetermined value of LC_50_ calculated previously [21]. The experiment was conducted by employing a semistatic system. At the end of exposure periods, liver tissue was removed and stored at -40°C for analysis.

### 2.2. Chemical Analysis of Fish for Cadmium Accumulation

Cadmium concentrations were measured directly in digested filtrates by Zeeman Atomic Absorption Spectrometry (Z-500) by following method #3500-Cd B of A.P.H.A. (2005) by process of wet digestion. 0.5 g of samples of fish organs, i.e., liver, heart, and skin, were 100 mL beakers and digested in *V*/*V* 3 : 1 composition of concentrated nitric acid and hydrochloric acid. The filtrates were analyzed for cadmium concentration on Zeeman Atomic Absorption Spectrometry (Z-500).

### 2.3. Qualitative and Quantitative Histological Assessment

Liver tissues of *C. idella* after cadmium exposure were randomly sampled for histopathological studies. The qualitative and quantitative assessment was carried out by analyzing the frequency, prevalence percentages, and histological alteration indices calculated by assessing histological alterations and comparison between the degrees of damage of the alterations in the same organ [22]. The identified individual alterations were given an importance factor according to the [23] that represented the intensity of the alterations to harm fish health. The score value and importance factor for each alteration were multiplied to find out the histological alteration index (HAI) values to calculate the degree of tissue damage by liver indices.

### 2.4. Total RNA Extraction and Preparation of cDNA

Liver tissue of 50 mg of grass carp *C. idella* was used for preparation of cDNA and extraction of total RNA for analysis of genes (metallothionein, heat shock proteins, and housekeeping gene B2M) expressions. Total RNA was extracted using a standard TRIzol procedure (Invitrogen) according to manufacturer's instructions. The DNA extraction kit was used for synthesis of cDNA according to the manufacturer's instructions. The purity of total RNA extracted and synthesized during the present study was checked and examined by agarose gel electrophoresis in which samples were run on 3% agarose gel to avoid disruption of bands. There was no or negligible degradation of total RNA during preparations and purification of samples. The samples were analyzed and amplified by using PCR technique by following the method of [24]. PCR was performed by the synthesis of primers for magnifications of heat shock proteins (HSP70), metallothionein (MT) genes, and housekeeping gene B2M (Table 1) calculated on the basis of specifically designed genomic DNA and sequence information of MT and HSP of *C. idella.* Housekeeping gene B2M was used as an internal control to normalize mRNA expressions in the PCR.

### 2.5. Statistical Analysis

All the data were presented as mean ± S.D. The histological alterations were observed by using microscope and photographed through an OPTIKA microscope. SPSS Ver. 21 statistical software was used for analysis and descriptive statistics to represent biometric data, HAI values, C.F. of control and treated groups to calculate the percentage prevalence for the number of fish that demonstrated with the same histological alterations.

## 3. Results

### 3.1. Fish Meat Quality Indicators and Specimen Data

The mean value of body mass (*w*), length (*L*), and condition factor of control fish were 10.00 ± 0.90 g, 9.20 ± 0.24 cm, and 1.30 ± 0.34 g cm^−3^, respectively, for the control fish whereas the condition factor of exposed fish depicted significantly lower value of 0.80 ± 0.34 g cm^−3^ as compared to control fish. The body length and body weight of exposed fish were 10.20 ± 0.69 cm and 9.20 ± 0.25 g, respectively. The condition factor of control fish was higher (1.30 ± 0.034 g cm^−3^) as compared to the exposed fish which showed better quality and taste of fish while lower mean value of condition factor of exposed fish (0.80 ± 0.34 g cm^−3^) indicated deteriorated meat quality and condition due to toxicity of cadmium presented in Figure 1.

### 3.2. Bioaccumulation of Cadmium in Fish Tissues

Control and exposed fish were compared for cadmium accumulation in different organs.  Figure 2 shows the metal accumulation levels in the liver, heart, and skin during chronic cadmium exposure. The accumulation values of cadmium in control carp fish were considerably low, but metal-exposed fish showed maximum value of accumulation. The mean value of cadmium in the liver of exposed fish, grass carp, was significantly high (1.78 ± 1.04 *μ*g g^−1^). The heart of the Cd-exposed fish accumulated cadmium with the mean value of 1.60 ± 0.05 *μ*g g^−1^ whereas the skin of the fish accumulated higher cadmium concentration (2.00 ± 0.04 *μ*gg^−1^).

### 3.3. Histological Assessment of Fish (*C. idella*)

Control fish liver represented particular parenchymatous appearance. The size and shape of the liver were normal for the unexposed fish (Figure 3(a)) whereas the exposed fish showed mild to severe lesions in the tissue structure, i.e., hypertrophy, vacuolar degeneration, hepatic necrosis, and dilated sinusoids (Figures 3(c)–3(e)).

Table 2 demonstrates the highest prevalence percentage of 90% observed for dilated sinusoids while the lowest prevalence percentage of 67% was recorded for partial degeneration of hepatic mass. In case of cadmium-exposed fish, the value of prevalence percentage was the highest (93%) for hemorrhage and 63% was the lowest value for proliferation of hepatic cells (Table 2). The prevalence percentage for diluted sinusoids was 60% and 90% for chronic exposure groups, respectively.  Table 3 shows comparison of semiquantitative scoring of histological changes in the liver of 28-day exposed fish and control (unexposed fish) and pronounced abrasions were hepatic necrosis, hyperplasia, hemorrhage, hepatic infiltration, dilated sinusoids, pyknotic nuclei, edema, fat cell accumulation, and hypertrophy.

The analysis of histological alteration indices (HAI values) depicted that mean HAI value for the liver of 28-day-treated fish was 78. Mean HAI value for focal area of necrosis and vacuolar degeneration was the highest as compared to other individual alterations, and it was reported as 9 whereas proliferation of hepatocytes showed mean HAI value of 2 under the same exposure conditions (Table 4).

The organ index (*I*_org_) of the liver tissue was calculated and described in Figure 4. The overall assessment of lesions found in liver tissue based on score and importance factor was 48. The comparison of reaction indices of various reaction patterns in liver tissues showed the highest reaction index for reaction pattern of regressive change was 32 while the lower organ index for reaction pattern of progressive change was observed as 8.

### 3.4. Changes in mRNA Expression Levels of Immune-Related Metallothionein and HSP70 under Sublethal Cadmium Exposure

The results of transcriptional levels of both genes were compared with housekeeping gene B2M transcriptional levels used as an internal control in liver samples of *C. idella* exposed to sublethal (1.495 mg L^−1^) concentration of cadmium. A fragment of housekeeping gene BM2 with a molecular weight of 46440.17 Da was cloned and amplified using primers specially designed for cloning and amplification. The product of 150 bp of housekeeping gene was utilized as an internal control for the analysis of relative expression of metallothionein (MT) and heat shock proteins (HSP70) during cadmium exposure. Housekeeping gene during the present investigation served as mediator for the evaluation mRNA expressions, processes of nucleic acid extraction and depiction PCR quality and quality of liver samples obtained from exposed fish. All the samples of liver showed higher value of relative abundance of mRNA expressions for metallothionein gene (*p* < 0.05) as shown in Figure 5. The molecular weight of metallothionein analyzed from the expressed transcriptional levels in the samples was 55892.06 Da. The metallothionein expression was compared and analyzed with a ladder consisting of 50 bp with lower and upper base pair sequences of 30 bp and 50 bp, respectively.

In the present investigation, expression analysis of HSP70 (a product of 107 base pairs) isolated from the liver samples exposed to sublethal cadmium concentrations revealed a molecular weight of 32805.14 Da. The fragments of cDNA in lanes 1 and 5 showed the ladder and housekeeping gene sequences, respectively. The sequences of HSP70 were expressed in lane 2-4 are amplified by using HSP70 reversed and forward sequences and revealed to be about 107 base pairs (bp) examined on the 3% agarose gel. The interrelation of transcriptional levels and cadmium retention in the liver of exposed grass carp attained the maximum (3.5 fold, *p* < 0.05) in the Cd-treated fish samples as compared to the control. The comparison of transcriptional levels of HSP70 and MT revealed that mRNA expressions of metallothionein gene were statistically significantly higher compared to the heat shock proteins. The analysis levels of expression of both genes (metallothionein and heat shock proteins 70) in the livers of treated fish exhibited higher expressions than housekeeping gene B2M. The expression levels of all the genes analyzed during the present investigation followed the order of magnitude as HSP > MT > B2M.

## 4. Discussion

Heat shock proteins have demonstrated the capacity of inducing the long-lasting protective immune responses and HSPs have been considered as proinflammatory damage-associated molecular response especially HSP60 and HSP70 [25, 26]. In the present investigation, the adaptive immune response of freshwater fish *C. idella* was studied by investigating the differential expression levels changes of HSP and MT genes exposed to cadmium toxicity.

The most important environmental problems are heavy metal pollution that leads to adaptive evolution of immune proteins in animals. The heavy metal toxicity induces changes in the expression levels of HSP and MT gene. The heavy metals released from industrial, man-made activities, domestic processes, and anthropogenic have adversely contaminated the aquatic systems. Heavy metal pollution has disturbing effects on the ecological balance of the environment. The most toxic heavy metal is cadmium and toxic for aquatic life as an environmental pollutant. After the maximum level of metals in the polluted aquatic system fish start collection of metals directly from the environment [27, 28]. The cadmium contamination of aquatic ecosystems has increased cadmium deposits in tissues of aquatic organisms in all food chains [29, 30].

The treated exposed to sublethal dose of cadmium exhibited a range of abnormal behavior consisting of restlessness, irregular movement patterns, slow feeding, lack of balance, erratic swimming, air gulping, excessive secretion of mucus, rolling movement, and swimming in the backward direction. Similar behavioral changes were also observed by [31], while control fish established normal physiology with no distinct behavioral changes. There was no physical change like fin rot, dropsy, itching, no tumors, and lesions in control fish. The behavioral changes seen are symptomatic of internal disturbances of the body functions such as inhibition of enzymes, impairment of neural transmission, and disturbances in metabolic pathways stated by Altindag [32]. The abnormal behavioral manifestations revealed by the fingerlings on contact to lead are similar to that reported for other toxicants like cadmium and chromium explained by [33].

During present studies, cadmium concentration demonstrated the deteriorated condition of fish, bioaccumulation of metal in heart, skin, and liver tissues, and histological alterations in the liver of fish exposed to Cd-contaminated medium. The mean value of condition factor of control fish as compared to exposed fish highlights poor condition and deteriorated meat quality of the fish due to cadmium exposure. The mean condition factor of fish for the control and exposed group was 0.7 ± 0.2, 0.8 ± 0.2, and 0.8 ± 0.2 g cm^−3^, respectively, recorded by [34]. The results of present investigation are also in accordance with McHugh [35]. Nonsignificant effects of Cd on rainbow trout, fathead minnow, and channel catfish are reported by [36]. Under metallic toxicity, rainbow trout showed reduced growth and lower FCE was due to slow rate of feeding; similarly, studies on the effect of chronic sublethal zinc exposure demonstrated growth inhibition in *Cirrhinus mrigala* [37].

Cadmium is a common heavy metal of natural waters and is highly toxic to the aquatic organisms even at very low concentration that can result into significantly lower condition factor indices in the exposed fish as observed during present investigation [38]. Effects of metallic toxicity on feed intake, growth, FCE, and condition factor of tilapia with decreased in meat quality interpreting it unhealthy for human consumption were reported by [39]. [40] also reported significantly decreased body condition factor and growth parameters of fish exposed to different concentrations of cadmium (*p* < 0.05) as compared to the control due to increase in stress as a result of cadmium exposure.

In the present investigation, the mean cadmium level in the liver of exposed fish (0.37 ± 0.027) was expressively higher compared to control fish. Perera et al. [41] reported higher concentration of cadmium in exposed fish liver when compared with control fish. The accumulation of metal in the liver of control and exposed fish was 12.4 and 82.1 mg/kg, respectively, and maximum metal accumulation in exposed fish as compared to control fish revealed negative impact of metals on tissues described by [42].

In the present investigation, the skin of the control fish revealed significantly lower mean cadmium concentration whereas the exposed fish accumulated cadmium with the mean value of 14.46 ± 41.65 mg L^−1^. The difference between the control and exposed fish for the accumulation of cadmium in the liver, heart, and skin remained significantly higher which showed negative impact of cadmium on fish body organs. The analysis of cadmium level in the tissues under the chronic exposure condition followed the order skin > liver > heart. Abdel-Warith et al. [43] reported that the higher accumulation of heavy metal in the liver may alter the level of various biochemical parameters and may also cause severe liver damage. Similar results were demonstrated by [44]. Malik et al. [45] reported that the concentration of heavy metals in liver of *L. rohita* and *C. straitus* was found to be higher than the other organs because the liver acted as an important organ for storage and detoxification.

The liver is a vital organ which is mostly affected by water pollutants because of its role in detoxification and biotransformation processes. After acute and chronic cadmium exposure, the histological alteration in the liver of *Ctenopharyngodon idella* was hemorrhage, edema, hypertrophy, hyperplasia, and hepatic cell necrosis. Ptashynski et al. [46] and Fanta et al. [47] described these alterations in fish liver by pollutants. *Clarias gariepinus* was exposed with lead and determined the degeneration of hepatocytes and focal area necrosis in the liver of fish by [48].

In the current investigation, the liver of exposed fish showed histopathological alteration such as hypertrophy, hyperplasia, necrosis, dilated sinusoids, inflammation, hemorrhages, pigmented cell rupture, focal area of necrosis, partial degeneration of hepatic mass, pyknotic nuclei, and congestion of central vein. The results are in accordance with [49] who described the similar histological alterations in the liver of fish, *Channa punctatus*, due to toxicant exposure. Progressive changes in the liver of exposed fish were hypertrophy, hyperplasia (enlargement of tissue by greater number of cells without change in volume of cells), and dilated sinusoids reported by the present study. In the present study, histological changes of desired organ investigated and pathological alterations determined during acute and chronic exposure of cadmium were explained into five major reaction patterns for assessment of histopathological alteration in exposed fish. According to the Wang et al. [17], Wang et al. [18], cadmium exposure caused histopathological changes in the liver and induced negative impact on immunity, stress defense mechanism, and metal transport system in grass carp (*Ctenopharyngodon idella*).

In the current study, the samples showed significantly increased expression of metallothionein gene due to cadmium accumulation and detoxification role performed by the liver. The analysis of relative abundance and transcriptional concentrations of metallothionein showed heightened levels in cadmium treated liver specimens as compared to the mRNA expression in the housekeeping genes as an internal control. The quantity of metallothionein gene expression in the liver varied significantly, and an initial 1.5-fold increase was observed due to toxic cadmium exposure and later it was magnified up to 3.5-fold showing direct dependence on the exposure duration and rate of cadmium accumulation in the liver of grass carp. [50] reported upregulated metallothionein expression levels in Cd-exposed fish due to accumulation of cadmium in the liver tissue suggestive of the cadmium toxicity effect on the regulation of gene transcription. The results are also in accordance with the study of [19, 21] who reported the effect of different absorption of cadmium was observed on tissue MT mRNA transcript level and showed that MT mRNA expression was definite and dose dependent on tissues of *Channa punctata*.

Different species of fish were used for observing the behavior of HSP70 in stress and unstressed cell. The heat shock cognate protein (HSC70) performed the different functions like formation of complex receptor, activin growth factor activation, and activation of morphogenetic protein of bone. Under stressed and normal condition, HSP70/HSC70 moved toward lysosomes which speed up protein degradation and catabolism [51].

In the present investigation, the analysis of HSP70 (a product of 107 base pairs) isolated from the liver samples revealed a molecular weight of 32805.14 Da. All the amplification products were similar to the corresponding genomic sequence of heat shock proteins. HSP levels have been reported to be associated with the environmental stress conditions mainly involved in the cellular defense pathways and detoxification mechanisms [16, 52–54]. Cadmium exposure induced the upregulation of HSP70 and MT expressions in aquatic organisms in several studies reported by Yu et al. [55]; Sung et al. [56]; Chung et al. [57]; Maulvault et al. [58].

The amount of relative abundance of mRNA showed significant increase as a result of 28-day exposure period. The expression of MT and HSP70 genes in Cd-stressed fish depicted clearly that fish exhibited stress-dependent pattern of mRNA expressions following the sublethal cadmium exposure. The same increasing trend was observed for all genes in all the examined fishes. The present study revealed higher upregulation of expression of HSP70 due to stressed culture conditions and higher rate of accumulation in fish organs causing impairments in gene regulation mechanisms. [28] also investigated the immune responses and changes in the expression of immune-related genes in the liver tissue of fish after sublethal cadmium exposure of 28 days. They confirmed the upregulation of HSP60, HSP70, and HSP90 indicative of cadmium-induced cellular stress. Very little information is available regarding the immunotoxicity of heavy metals in the metal-exposed fish at the gene level. Therefore, we evaluated the immunotoxicity of cadmium and changes in the expression levels of immune-related genes and reported the quantity of relative expression of metallothionein (MT) and heat shock proteins increased with an increase in rate of cadmium accumulation under laboratory conditions. The same results were reported by Safari et al. [59] when juveniles of Persian sturgeon were used for determining mRNA-HSP70 expression in the liver and gills after 14-day exposure of sublethal doses of CdCl_2_ (0.05, 0.1, and 0.2). HSP70 was cloned from liver cell of fish having 72-nucleotide fragment. The expression level of mRNA-HSP70 was increased (*p* ≤ 0.05) in the tissues of the liver and gills of exposed fish when compared with control. [60] also reported the immunotoxicological effect of metals and [61, 62] revealed an increase in the HSP70 due to the overexpression of HSP70. In conclusion, it is confirmed from the present study that tissue stress resulting from the inflammation and toxicity exposure causes upregulated levels of intracellular HSPs and MT genes and may act as functional biomarker of evaluating the impact of toxicants on the immune responses of animals specifically HSP70 as a key regulator. So, the gene expression changes of immune-related proteins (HSP70 and MT) in exposed fish liver after chronic toxicity can be used a diagnostic tool of stress conditions and effect on the immune proteins.

## Figures and Tables

**Figure 1:** Mean values of body mass, body length, and condition factor of control and treated fish for visual health assessment.

**Figure 2:** Bioaccumulation of cadmium in the liver, skin, and heart of fish after cadmium exposure.

**Figure 3:** Photomicrograph of liver of fish: (a) control fish; (b–d) under cadmium exposure showing V: vessels; S: sinusoids; HC: hepatic cells; BH: blood damage; NC: necrosis; HH: hypertrophy; HV: hepatic vacuoles; Hae: hemorrhage (4 *μ*m thick; H&E staining; 10x).

**Figure 4:** Calculation of reaction indices in the liver of fish exposed to sublethal cadmium levels.

**Figure 5:** Comparison of mRNA expression of metallothionein, heat shock proteins (HSP70), and beta-2-microglobulin (B2M) due to cadmium dose kinetics under sublethal exposure conditions.

**Table 1:** List of primers used for the heat shock proteins (HSP70), metallothionein (MT), and beta-2-microglobulins (BM2), melting temperature (Tm).

Gene	Forward and reverse sequence	Tm	GC content (%)	3′ complementarity	Product
HSP	Primer F: CTGCTGGATGTGGCTCCTCTGTC	64.96	60.8764.96	1.00	107
	Primer R: AAGGTCTGGGTCTGTTTGGTGGG	64.51	56.52	0.00	
MT	Primer F: ATGGATCCTTGCGATTGCG	58.68	52.63	2.00	182
	Primer R: CATTGACAGCAGCTGGAGCC	61.65	60.00	4.00	
B2M	Primer F: GGCTGGCAGTTTCACCTCAC	61.52	61.52	0.00	150
	Primer R: CCACCCTTTGTCTGGCTTTG	59.32	55.00	0.00	

**Table 2:** Frequency and prevalence percentage of histological alteration of *Ctenopharyngodon idella* exposed under acute and chronic toxicity of cadmium.

Organ	Histological alterations	Frequency (*n* = 30)	Prevalence (%)
Liver	Nuclear alteration	**22**	**73**
	Hepatic necrosis	**26**	**87**
	Hyperplasia	**25**	**83**
	Hemorrhage	**28**	**93**
	Hepatic infiltration	**23**	**77**
	Dilated sinusoids	**27**	**90**
	Cognation of central vein	**20**	**67**
	Pyknotic nuclei	**22**	**73**
	Proliferation of hepatic cells	**19**	**63**
	Edema	**23**	**77**
	Pigmented cell rupture	**21**	**70**
	Fat cell accumulation	**24**	**80**
	Hypertrophy	**25**	**83**
	Alarm cells	**19**	**63**
	Partial degeneration of hepatic mass	**20**	**67**
	Vacuole degeneration	**25**	**83**

**Table 3:** Histological alterations in the liver of *Ctenopharyngodon idella* determined by using semiquantitative scoring method.

Histological alterations	Control	Cd-exposed group
Nuclear alterations	−	++
Hepatic necrosis	−	+++
Hyperplasia	−	+++
Hemorrhage	−	+++
Hepatic infiltration	−	+++
Dilated sinusoids	−	+++
Cognation of central vein	−	++
Pyknotic nuclei	−	+++
Proliferation of hepatocytes	−	++
Edema	−	+++
Pigmented cell rupture	−	++
Fat cell accumulation	−	+++
Hypertrophy	−	+++
Alarm cell	−	++
Partial degeneration of hepatic mass	−	++
Vacuole degeneration	−	+++

Results of histological assessment evaluated as mild and minor abrasions ≤ 25% represented by +; medium abrasions ≤ 50% represented by ++; pronounced abrasions ≤ 75% represented by +++; severe abrasions ≥ 75% represented by ++++, and no histological alteration ≤0% represented by −.

**Table 4:** HAI index assessment of the liver of exposed *Ctenopharyngodon idella* by using importance factor and score value of cadmium chronic toxicity.

Histological abrasions	Importance factor (*w*)	Score value (*a*)	Index (*I*)	HAI (*a* × *W*)
Hemorrhage	*W*_lC1_ = 1	*a*_IC1_ = 3	I_IC_	3
Edema	*W*_lC2_ = 2	*a*_IC2_ = 3		6
Hepatic necrosis	*W*_IRI_ = 3	*a*_IR1_ = 3	*I*_IR_	9
Partial degeneration of hepatic mass	*W*_IR2_ = 1	*a*_IR2_ = 2		2
Congestion of central vein	*W*_IR3_ = 2	*a*_IR3_ = 2		4
Vacuole degeneration	*W*_IR4_ = 3	*a*_IR4_ = 3		9
Alarm cells	*W*_IR5_ = 1	*a*_IR5_ = 2		2
Focal area of necrosis	*W*_IR16_ = 3	*a*_IR16_ = 3		9
Dilated sinusoids	*W*_IP1_ = 3	*a*_IP1_ = 3	I_IP_	9
Pigmented cell ruptured	*W*_II1_ = 2	*a*_II1_ = 2		4
Fat cell accumulation	*W*_II2_ = 1	*a*_II2_ = 3		3
Hyperplasia	*W*_LP4_ = 2	*a*_LP4_ = 3	*I*_LP_	6
Hypertrophy	*W*_LP5_ = 1	*a*_LP5_ = 3		3
Hepatic infiltration	*W*_II3_ = 1	*a*_II3_ = 3		3
Nuclear alteration	*W*_LR16_ = 2	*a*_LR16_ = 2	*I*_LR_	4
Proliferation of hepatocytes	*W*_LI3_ = 1	*a*_LI3_ = 2	*I*_LI_	2
Mean value of *I*_liver_				78

## Data Availability

The data used to support the findings of this study are included within the article.
